# Haemin attenuates intermittent hypoxia‐induced cardiac injury via inhibiting mitochondrial fission

**DOI:** 10.1111/jcmm.13560

**Published:** 2018-03-07

**Authors:** Qian Han, Guihua Li, Mary SiuMan Ip, Yuelin Zhang, Zhe Zhen, Judith ChoiWo Mak, Nuofu Zhang

**Affiliations:** ^1^ State Key Laboratory Guangzhou Institute of Respiratory Health Department of Respiratory Medicine The First Affiliated Hospital of Guangzhou Medical University Guangzhou China; ^2^ Li Kashing Faculty of Medicine Department of Medicine The University of Hong Kong Hong Kong China

**Keywords:** apoptosis, fission, haeme oxygenase‐1, haemin, intermittent hypoxia, mitochondria

## Abstract

Obstructive sleep apnoea (OSA) characterized by intermittent hypoxia (IH) is closely associated with cardiovascular diseases. IH confers cardiac injury via accelerating cardiomyocyte apoptosis, whereas the underlying mechanism has remained largely enigmatic. This study aimed to explore the potential mechanisms involved in the IH‐induced cardiac damage performed with the IH‐exposed cell and animal models and to investigate the protective effects of haemin, a potent haeme oxygenase‐1 (HO‐1) activator, on the cardiac injury induced by IH. Neonatal rat cardiomyocyte (NRC) was treated with or without haemin before IH exposure. Eighteen male Sprague‐Dawley (SD) rats were randomized into three groups: control group, IH group (PBS, ip) and IH + haemin group (haemin, 4 mg/kg, ip). The cardiac function was determined by echocardiography. Mitochondrial fission was evaluated by Mitotracker staining. The mitochondrial dynamics‐related proteins (mitochondrial fusion protein, Mfn2; mitochondrial fission protein, Drp1) were determined by Western blot. The apoptosis of cardiomyocytes and heart sections was examined by TUNEL. IH regulated mitochondrial dynamics‐related proteins (decreased Mfn2 and increased Drp1 expressions, respectively), thereby leading to mitochondrial fragmentation and cell apoptosis in cardiomyocytes in vitro and in vivo, while haemin‐induced HO‐1 up‐regulation attenuated IH‐induced mitochondrial fragmentation and cell apoptosis. Moreover, IH resulted in left ventricular hypertrophy and impaired contractile function in vivo, while haemin ameliorated IH‐induced cardiac dysfunction. This study demonstrates that pharmacological activation of HO‐1 pathway protects against IH‐induced cardiac dysfunction and myocardial fibrosis through the inhibition of mitochondrial fission and cell apoptosis.

## 1 INTRODUCTION

Obstructive sleep apnoea (OSA) is characterized by recurrent episodes of airway collapse leading to intermittent hypoxia (IH) during nocturnal sleep. OSA has become a heavy medical burden worldwide because it is a critical risk factor for cardiovascular diseases.^1^, ^2^, ^3^, ^4^ Accumulating evidence has demonstrated that IH leads to cardiac injury through regulating mitochondrial function.^5^, ^6^ Indeed, cardiomyocytes hold a huge number of mitochondria to provide the ATP production for maintaining cardiac function. Mitochondria dynamics characterized by fusion and fission mediates the cell function.^7^, ^8^ Mitochondria fusion, regulated by the proteins mitofusin 1 (Mfn1) and Mfn2, leads to mitochondria elongation to protect the cell function.^9^, ^10^ On the contrary, mitochondria fission mediated by cytosolic protein dynamin‐related protein 1 (DRP1) and mitochondrial fission 1 (Fis1) results into mitochondrial fragmentation, and therefore inducing cell apoptosis.^11^, ^12^ The mitochondrial fusion and fission keep in balance to maintain mitochondrial function. Under pathologic conditions, mitochondrial fission outweighs fusion and leads to cardiomyocyte apoptosis and subsequent heart failure.^13^ Nevertheless, it has not been determined whether IH induced cardiac injury via regulating mitochondrial dynamics, that is fusion and fission.

Haeme oxygenase‐1 (HO‐1), an inducible stress response gene, degrades haeme into carbon monoxide (CO), free iron and biliverdin.^14^ HO‐1 has been intensively investigated and shown promising results in cellular protection on cardiovascular diseases via acting as an antioxidant, anti‐inflammatory and anti‐apoptotic system.^14^, ^15^ IH was shown to up‐regulate hepatic HO‐1 expression, thereby limiting hepatic pathogenesis in rats fed a high‐fat diet.^16^ On the contrary, the protective effect of IH‐induced HO‐1 was not observed in heart tissue as we previously found that the compensated HO‐1 up‐regulation induced by IH was not sufficiently able to attenuate the cardiomyocyte apoptosis and cardiac injury in rats.^17^ This was in agreement with other study showing the occurrence of heart failure with coronary ligation in mice albeit with enhancement of cardiac HO‐1 expression.^18^ On the other hand, haemin‐induced HO‐1 elevation was found to greatly inhibit cell apoptosis induced by IH in endothelial cells,^19^ yet the underlying mechanisms are yet to be demonstrated. It was reported that HO‐1 overexpression protects doxorubicin‐induced dilated cardiomyopathy via inhibiting Fis1 and increasing Mfn1/Mfn2 expression, suggesting that HO‐1 plays a critical role in mediating mitochondrial dynamics to regulate heart function.^20^

Based on these findings, we have been suggested that IH could disturb mitochondrial dynamics via inducing mitochondrial fission, thereby leading to cardiomyocyte apoptosis and cardiac dysfunction. Haemin, an HO‐1 inducer, could attenuate IH‐induced cardiac dysfunction through the inhibition of mitochondrial fragmentation and cardiomyocyte apoptosis.

## 2 MATERIALS AND METHODS

### 2.1 Isolation and culture of neonatal rat cardiomyocyte (NRC)

The NRCs were isolated as previously described.^21^ The isolated NRCs were plated on the in 24‐well plates containing collagen‐coated glass coverslips or 6‐well plates at a density of 2  ×  10^5^ cells/mL and then cultured under the normoxia or IH exposure according to the experimental requirements.

### 2.2 IH‐exposed cell culture model and treatment

IH‐exposed cell culture model was established as previously reported.^19^ Briefly, when NRCs achieved 80%‐90% confluency, NRCs were treated with 1% FBS medium for 24 hours for starvation before different treatments. For IH exposure, cells were cultured in an incubator chamber with 5% CO_2_ connected to BioSpherix OxyCycler (Biospherix, Redfield, NY, USA) and controlled by a custom‐designed computer. The O_2_ levels were set up by 1% for 10 minutes and 21% for 5 minutes. We performed 64, 96 and 128 cycles of IH in the pilot study and found that IH treatment for 96 cycles induced maximum apoptosis without significant cell death (data not shown). Cells were therefore exposed to normoxic or IH for 96 cycles for interventional study (approximately 27 hours). Cells were cultured in normoxic condition as the negative control group (21% O_2_ and 5% CO_2_) throughout the same period of exposure. For haemin treatment, haemin dissolved in dimethyl sulfoxide (DMSO) was added into the medium to give a final concentration of 10 μM at 30 minutes before IH exposure. An equal volume of DMSO was added to cells as controls.

### 2.3 Transfection

Control siRNA or HO‐1 siRNA (50 nM) was transfected performed with RNAiMax (Invitrogen) according to protocol. Briefly, NRCs were cultured to 70%‐80% confluence prior to transfection. The siRNA transfection reagent mixture was prepared and then added into NRCs. Cells were then incubated for 24~48 hours, and the transfected efficiency was determined by Western blot.

### 2.4 Mitochondrial staining

Mitochondrial staining was performed as previously described.^8^ Briefly, NRCs were plated on the cover slips. After treatment, NRCs were stained with 0.01 μM MitoTracker^®^ Green FM (M7514, Thermo Fisher Scientific) for half hour. After washed with PBS, NRCs were mounted with DAPI and then imaged by a laser scanning confocal microscope. Six fields were randomly observed and counted. The percentage of fragmented mitochondria was calculated by the cells with fragmented mitochondria to the total number of cells.^8^

### 2.5 Animal experiment

All experiments with animals in this study were approved by the Committee on the Use of Live Animals in Teaching and Research of the University of Hong Kong (CULTAR 2371‐11). Male Sprague–Dawley rats weighing 150~200 g were housed in a temperature‐controlled atmosphere, 12/12‐hour light/dark cycle and given free access to food and water. The rats (n = 18) were randomly divided into 3 groups: control group (n = 6), IH group (n = 6) and IH + haemin group (n = 6). Rats were received the intraperitoneal injection of PBS in the IH group or haemin (dissolved in 0.1M sodium hydroxide) at a dose of 4 mg/kg body weight every other day before exposure to IH protocol (IH + haemin group) as previously reported.^17^ Haemin dose was selected on the basis of a previous study.^22^ The IH procedure was repetitive 4 minutes 10% O_2_ and 2 minutes 21% O_2_ for 8 hours per day for 6 weeks. In the control group, the rats were received intermittent air at the same flow rate. Six weeks after treatment, the cardiac function was measured by echocardiography, and subsequently, all the rats were killed, and then, hearts were harvested for further analysis.

### 2.6 Histological analysis

The hearts of rats were collected, fixed, embedded and finally sectioned into 5‐μm slides. Fibrosis formation was evaluated by sirius red staining. The degree of fibrosis was analysed by two independent investigators and expressed as a percentage of the whole heart. The size of the fibrotic area was quantified with 6 randomly chosen high‐power fields for each heart section, 6 rats for each group.

### 2.7 Western blot

The cells and heart tissue proteins were extracted in lysis buffer supplemented with a protease inhibitor, and then, the concentration was measured. Besides, mitochondrial protein was extracted performed with Cytosol/Mitochondria Fraction Kit according to the manufacturer's instruction (Calbiochem, MA, USA). Subsequently, the proteins were resolved on SDS‐PAGE, transferred to PVDF membranes and then incubated with the primary antibodies overnight at 4°C. The primary antibodies were listed as following: HO‐1 (Abcam, MA, USA), Mfn2, Drp1 (Santa Cruz Bioechnology, Texas, USA), cleaved caspase‐3, caspase‐3, Bax, Bcl2 (Cell Signalling, Danvers, MA, USA). The membranes were later incubated with horseradish peroxide‐conjugated goat anti‐rabbit, goat antimouse or mouse anti‐goat antibody (Dako, Danmark) for 2 hours at room temperature. Afterwards, membranes were probed with enhanced chemiluninescence (ECL plus) (Amersham, Piscataway, UK). GAPDH and β‐actin (Santa Cruz) were used as loading control for in vivo and in vitro experiment, respectively, and mitochondrial protein was normalized to Cox 4 (Abcam). Desitometric analysis of the bands was performed with GeneTools (Syngene), and results were expressed as fold change to relative control.

### 2.8 TUNEL assay

The apoptosis of cardiomyocytes was examined by terminal deoxynucleotidal transferase‐mediated dUTP nick end‐labelling (TUNEL) staining in accordance with the kit instructions (11684795910, Roche). Briefly, after washing with PBS, NRCs or heart sections were incubated with 1 μg/mL Proteinase K/10 mM Tris solution for 15 minutes at room temperature. Subsequently, the sections or NRCs were washed twice in PBS and then incubated with the TUNEL reaction mixture at 37°C for 1 hour. Finally, sections or NRCs were washed with PBS twice, mounted with DAPI and photographed performed with a fluorescent microscope. Five sections were randomly collected from each rat, and six rats from each group were analysed.

### 2.9 Caspase‐3 activity

The heart tissue was homogenized and centrifuged at 15 000 *g* for 5 minutes, and the supernatant was fivefold diluted with the homogenizing medium previously described. A 150‐μL aliquot of this mixture was assayed performed with the commercial kit—Caspase‐3 assay kit, Fluorimetric^®^ (CASP3F, Sigma, St Louis, MO, USA), according to the manufacturer's instructions.

### 2.10 Statistical analysis

Data are shown as the mean ± SEM of at least three independent experiments. One‐way ANOVA test followed by Bonferroni test was applied to analysis of multiple groups and, unpaired Student's *t* test was applied to compare two groups. All the statistical analyses were performed using GraphPad Prism 5.0 (GraphPad Software Inc, San Diego, CA, USA), and a *P*‐value <.05 was considered statistically significant.

## 3 RESULTS

### 3.1 IH induces mitochondrial fission and cell apoptosis in cardiomyocytes

To test whether IH could induce mitochondrial fission and cell apoptosis, we treated NRCs with IH and then performed Mitotracker staining. The mitochondrial fragmentation was significantly increased in the IH group compared with the control group (Figure 1A‐i and ii). Meanwhile, compared with the control group, the expression level of Mfn2 was significantly down‐regulated whereas Drp1 was up‐regulated in the IH group (Figure 1B‐i, ii and iii). Furthermore, IH exposure resulted into a striking increase in the apoptosis in NRCs (Figure 1C‐i and ii). Taken together, these results show that IH induces mitochondrial fission and apoptosis in cardiomyocytes.

**Figure 1:** IH induces mitochondrial fission and cell apoptosis in cardiomyocytes. (A) Representative images showing the fragmented mitochondria in NRCs under control or IH exposure (i). The fragmented mitochondria induced by IH were counted (ii). Scale bar = 50 μm. (B) Western blot analysis for the expression of Mfn2 and Drp1 under control or IH exposure (i). The expression levels of Mfn2 (ii) and Drp1 (iii) among the different groups were evaluated. (C) Representative images showing the apoptosis of NRCs under control or IH exposure (i). The apoptosis of NRCs under control or IH exposure was analysed (ii). Scale bar = 50 μm. Data were presented as means ± SEM. **P < .01 vs Control

### 3.2 HO‐1 inhibits mitochondrial fission and apoptosis induced by IH in cardiomyocytes

The expression level of HO‐1 was greatly enhanced in response to IH exposure (Figure 2A‐i, ii); however, despite up‐regulation of HO‐1 under IH exposure, the increased HO‐1 did not ameliorate mitochondrial fission and cell apoptosis induced by IH in cardiomyocytes. To further determine the exact role of HO‐1 in the regulation of mitochondrial fragmentation, we treated NRCs with HO‐1siRNA and then exposed to IH. The increased HO‐1 induced by IH was abrogated in HO‐1siRNA‐treated NRCs (Figure 2B‐i and ii). Interestingly, mitochondria fragmentation and cell apoptosis were significantly increased in HO‐1siRNA‐treated NRCs compared with native NRCs exposed to IH (Figure 2B‐iii and iv). Thus, it appears that HO‐1 inhibits the mitochondrial fission and cell apoptosis induced by IH.

**Figure 2:** HO‐1 inhibits mitochondrial fission and cell apoptosis in cardiomyocytes. (A) The expressions of HO‐1 under control or IH exposure were determined (i) and evaluated (ii) by Western blot. (B) The protein expression levels of HO‐1 in NRCs from control, IH and IH + HO‐1siRNA groups were determined by Western blot (i) and evaluated by densitometry (ii). The fragmented mitochondria (iii) and the apoptosis of NRCs (iv) from control, IH and IH + HO‐1siRNA groups were analysed. Data were presented as means ± SEM. **P < .01 and ***P < .001 vs control, respectively; ^*##*^ *P *< .01 vs IH

### 3.3 Haemin attenuates mitochondrial fission and cell apoptosis induced by IH in cardiomyocytes

Haemin is an HO‐1 inducer, and we, thus, treated the NRCs with haemin and then exposed to IH to examine the functional role of haemin on IH‐induced mitochondrial fission and cell apoptosis in cardiomyocytes. Western blot showed that haemin‐treated NRCs displayed a significantly increased expression of HO‐1 under IH challenge compared with native NRCs (Figure 3A‐i and ii). The IH‐induced mitochondrial fragmentation was greatly reduced after haemin treatment (Figure 3B‐i and ii), and the expression of Mnf2 was markedly increased whereas the expression of Drp1 was notably decreased in the IH + haemin group compared with the IH group (Figure 3C‐i, ii and iii). Moreover, TUNEL showed that haemin treatment could greatly inhibit IH‐accelerated NRCs apoptosis (Figure 3D‐i and ii). Taken together, these results suggest that haemin attenuates IH‐induced mitochondrial fission and cell apoptosis in cardiomyocytes.

**Figure 3:** Haemin attenuates mitochondrial fission and cell apoptosis in cardiomyocytes. (A) The protein expression levels of HO‐1 in NRCs from control, IH and IH + haemin groups were determined by Western blot (i) and evaluated by densitometry (ii). (B) Representative images showing the fragmented mitochondria in NRCs from control, IH and IH + haemin groups (i). The fragmented mitochondria from different groups were counted (ii). Scale bar = 50 μm. (C) Western blot analysis for expression levels of Mfn2 and Drp1 in NRCs from control, IH and IH + haemin groups (i). The expressions of Mfn2 (ii) and Drp1 (iii) among the different groups were evaluated by densitometry. (D) Representative images showing the apoptosis of NRCs from control, IH and IH + haemin groups (i). The apoptosis of NRCs among the different groups was analysed (ii). Scale bar = 50 μm. Data were presented as means ± SEM. **P < .01 and ***P < .001 vs control, respectively; ^##^ *P *< .01 vs IH

### 3.4 Haemin effectively protects against IH‐induced cardiac injury

The experimental protocol is outlined in Figure 4A. Cardiac function among different experimental groups was evaluated by echocardiogram (Figure 4B‐i). The data from echocardiographic study are shown in Table 1. The left ventricular ejection fraction (LVEF), fractional shortening (FS) and LV internal diameter end diastole (LVIDd) were greatly reduced whereas LV posterior wall end diastole (LVPWd) was significantly increased in the IH group compared with the control group, indicating IH‐induced cardiac hypertrophy and contractile dysfunction in rats (Figure 4B‐ii). However, 6 weeks after haemin treatment, LVEF, FS and LVIDd were remarkably enhanced and LVPWd was reduced under IH exposure, suggesting that haemin ameliorates the cardiac dysfunction induced by IH (Figure 4B‐ii). Histological analysis revealed IH‐induced heart hypertrophy and haemin effectively attenuated heart hypertrophy (Figure 4C‐i). Sirius red staining showed a significantly enhanced extent of myocardial fibrosis in the IH group compared with the control group (Figure 4C‐ii and iii). Nonetheless, 6 weeks after haemin administration, myocardial fibrosis was remarkably decreased compared with the IH group (Figure 4C‐ii and iii). These results demonstrate that haemin effectively protects against IH‐induced cardiac injury.

**Figure 4:** Haemin effectively protects against IH‐induced cardiac injury. (A) Schematic diagram of IH exposure and haemin treatment. (B) Representative sonographic (M‐mode long‐axis) images of the heart in rats among the different groups (i). Cardiac function including LVIDd, LVPWd, LVEF and LVFS was measured in rats from control, IH and IH + haemin groups (n = 6 rats per group) (ii). (C) Histological analysis of heart sections from different groups stained with haematoxylin and eosin (H and E) (i). Scale bar = 2 mm. Sirius red staining demonstrated different degrees of fibrosis in the heart tissue among control, IH and IH + haemin groups (ii). Quantitative measurement of heart fibrosis in different experimental groups (iii) (n = 6). Scale bar = 100 μm. Data were presented as means ± SEM. *P < .05 and **P < .01 vs control, respectively; ^*#*^ *P *<* *.05 and ^*##*^ *P* < .01 vs IH, respectively

**Table 1:** Raw echocardiography values of rats from the different groups

	Control	IH	IH + haemin
LVIDd (mm)	8.78 ± 0.25	7.33 ± 0.23**	7.88 ± 0.21* ^,^ #
LVIDs (mm)	5.25 ± 0.2	4.69 ± 0.1**	4.78 ± 0.2*
LVPWd (mm)	1.67 ± 0.18	2.35 ± 0.1**	2.1 ± 0.11* ^,^ #
LVPWs (mm)	2.34 ± 0.2	2.69 ± 0.1**	2.59 ± 0.1*
EF (%)	74.6 ± 3.0	66 ± 2.1**	70.7 ± 2.5* ^,^ #
FS (%)	39.4 ± 1.7	33.4 ± 1.3**	36.5 ± 1.5* ^,^ #

LVIDd, left ventricular internal diameter end diastole; LVIDs, left ventricular internal diameter end systole; LVPWd, left ventricular end diastolic posterior wall dimension; LVPWs, left ventricular end systolic posterior wall dimension; LVEF, left ventricular ejection fraction; FS, fractional shortening.

Results are expressed as mean ± SEM; n = 5~6.

*P < .05 and **P < .01 vs control, respectively; ^*#*^ *P *< .05 vs IH.

### 3.5 Haemin ameliorates IH‐induced mitochondrial fission in rat heart via HO‐1

Subsequently, we explored whether haemin is involved in mediating the mitochondrial fragmentation via regulating HO‐1 in rats. First, we examined the expression of HO‐1 among different experimental groups. The expression of HO‐1 was dramatically increased in the IH + haemin group compared with the IH group (Figure 5A‐i and ii). Next, we examined the effect of haemin on mitochondrial fragmentation in the heart tissue. Compared with the IH group, the level of Drp1 was efficiently reduced while the level of Mfn2 was significantly up‐regulated in the IH + haemin group (Figure 5B‐i, ii and iii). These results support that haemin ameliorates IH‐induced mitochondrial fission in rats via the up‐regulation of HO‐1.

**Figure 5:** Haemin ameliorates mitochondrial fission induced by IH in rats via HO‐1. (A) Western blot analysis for the expression of HO‐1 in heart tissue from control, IH and IH + haemin groups (i). The expression levels of HO‐1 among the different groups were evaluated by densitometry (ii). (B) Western blot analysis for the expression of Mfn2 and Drp1 in heart tissue from control, IH and IH + haemin groups (i). The expression levels of Mfn2 (ii) and Drp1 (iii) among the different groups were evaluated by densitometry. Data were presented as means ± SEM. *P < .05, **P < .01 and ***P < .001 vs control, respectively; ^*##*^ *P *<* *.01 vs IH, respectively

### 3.6 Haemin attenuates IH‐induced apoptosis in rat heart tissue

Apoptosis of cardiomyocytes in the rat heart tissue among different groups was detected by TUNEL staining. As shown in Figure 6A, the apoptosis of cardiomyocytes was significantly enhanced in the IH group compared with the control group (Figure 6A‐i and ii). However, haemin treatment notably reduced the apoptosis of cardiomyocytes induced by IH (Figure 6A‐i and ii). Moreover, haemin treatment also attenuated IH‐induced elevation of caspase‐3 activity (Figure 6B), cleaved caspase3/caspase3 and Bax/Bcl‐2 expression (Figure 6C‐i and ii).

**Figure 6:** Haemin attenuates apoptosis induced by IH in rats. (A) Representative images showing the apoptosis of cardiomyocytes from control, IH and IH + haemin groups (i). The apoptosis of cardiomyocytes among different groups was analysed (ii). Scale bar = 100 μm. (B) Effect of IH/haemin on caspase‐3 activity in rat cardiac tissue. (C) Western blot analysis for the expression of Bax, Bcl‐2, cleaved caspase 3 and caspase 3 in heart tissue from control, IH and IH + haemin groups (i). The expression levels of Bx/Bcl‐2 (ii) and cleaved caspase 3/caspase 3 (iii) among the different groups were evaluated by densitometry. Data were presented as means ± SEM. *P < .05 and **P < .01 vs control, respectively; ^*#*^ *P *< .05 and ^*##*^ *P *< .01 vs IH, respectively

## 4 DISCUSSION

Over the past decades, OSA as an independent risk for cardiovascular diseases has attracted huge interest.^23^, ^24^, ^25^ Much attention has focused on the effect of IH, a characteristic pathophysiologic feature of repetitive obstructed breathing events. We found that the IH treatment resembling a moderate OSA condition led to left ventricular cardiac hypertrophy and contractile dysfunction, and the functional compromise was accompanied by structural impairment, that is interstitial fibrosis. These results are consistent with findings reported by us and other groups, showing IH‐induced ventricular remodelling and cardiac dysfunction.^5^, ^17^, ^26^, ^27^

Apoptosis constitutes one of the major mechanisms acting as intermediary pathogenic links between OSA and cardiovascular disorders. Cardiomyocyte apoptosis contributes to cell loss followed by progressive myocardial dysfunction and the eventual heart failure. Our previous study has shown that IH for 4 weeks could induce cholesterol accumulation in the rat heart and activate caspase‐dependent apoptosis, ultimately leading to myocardium damage.^17^ IH also stimulates pro‐apoptotic endoplasmic reticulum stress and thus increases myocardial infarct size.^26^ Despite encouraging results shown in some studies, the underlying mechanisms of IH‐induced cardiomyocyte apoptosis still have not been fully understood.

The heart is an organ that requires high energy to drive the blood flow. The energy is predominately provided by cardiac mitochondria which synthesis ATP via oxidative phosphorylation (Ox‐Phos).^28^ Therefore, cardiac mitochondria dysfunction contributes to the development of cardiovascular diseases including cardiovascular ageing,^29^ cardiomyopathy^28^ and cardiac hypertrophy.^30^ Mitochondria are dynamic organelles with constant fission and fusion. Once the balance of mitochondrial fission and fusion is disrupted, cardiomyocytes apoptosis consequently occurs and eventually leads to heart failure. Recent work has also shown that IH can cause mitochondrial abnormalities and myocardium interstitial fibrosis in apolipoprotein E‐knockout mice fed with high‐fat diet^27^; however, it is still unclear whether the imbalance of mitochondrial fission and fusion plays a role in the pathological change in cardiac tissue. In current study, we showed that IH treatment increased mitochondrial fragmentation and cell apoptosis in NRCs and rat heart tissue, which were associated with enhanced expression of Drp1 and reduced expression of Mfn2. Thus, our study indicates that IH‐induced mitochondrial fragmentation and subsequent cardiomyocyte apoptosis may underlie the important pathophysiological mechanisms in cardiac injury.

HO‐1 has generated much interest as a key biological molecule in the adaptation and/or defence against cellular stresses. Increasing evidence has demonstrated that HO‐1 possess protective effect on cardiovascular injury via suppressing oxidative stress,^15^ attenuating post‐ischaemic inflammation^31^ and inhibiting apoptosis.^32^ Recent studies also have shown that HO‐1 mediates the balance of the dynamic mitochondrial fusion and fission not only in the lung^33^ but also in the heart.^20^ HO‐1 overexpression protected the mice from doxorubicin‐induced dilated cardiomyopathy through regulating mitochondrial quality control, including the inhibition of Fis1 and the up‐regulation of Mfn1 and Mfn2.^20^ In our study, the up‐regulation of Drp1 and suppression of Mfn2 were accompanied by the increased expression of HO‐1 under IH exposure in vitro and in vivo, in contrast to the protective role of HO‐1 in mitochondrial integrity and function. However, it was also demonstrated by a previous study that coronary ligation to adult male mice resulted in left ventricular remodelling and dysfunction together with increased expression of HO‐1, indicating that the compensatory up‐regulation of HO‐1 may not sufficiently protect heart from various insults under such deleterious circumstances.^18^ Moreover, inhibition of HO‐1 performed with siRNA in NRCs greatly potentiated mitochondrial fragmentation and cell apoptosis induced by IH, further suggesting that the stimulation or overexpression rather than adaptive induction of HO‐1 may be capable of exerting cardiac protective effect.

Although several strategies, including positive airway pressure and telemedicine, are recommended to treat cardiovascular diseases in patients with OSA, the benefits are moderate.^1^, ^34^ Needless to say, exploring some novel therapies for these patients is urgently needed. Haemin has been reported to exhibit the cardioprotective effects by up‐regulating HO‐1 to exert pronounced anti‐inflammatory, anti‐oxidative as well as anti‐apoptotic activities.^22^ Haemin treatment was shown to decrease cardiac oxidative stress and intracellular fibrosis in a rat model of systemic hypertension.^35^ Pre‐treatment with haemin was found to protect the heart from post‐ischaemiac dysfunction and ventricular fibrillation in male Wistar rats.^36^ The cardioprotective effect of haemin was also demonstrated in our study showing that haemin treatment mitigated cardiac dysfunction and interstitial fibrosis induced by IH together with suppression of mitochondrial fission and cell apoptosis.

We have reported that haemin treatment could suppress the adverse effects of IH on oxidative stress and cell apoptosis in EAhy926 endothelial cells, although the underlying mechanisms were not fully illustrated in the previous study. Here, we found haemin treatment greatly increased HO‐1 expression, concomitantly suppressing mitochondrial fragmentation and cell apoptosis in NRCs as well as in a rat model of IH. Taken together with previous data of HO‐1 inhibition with siRNA in NRCs, our results suggested that haemin stimulated up‐regulation of HO‐1 and exerted the cardioprotective effect under IH exposure via, at least in part, targeting mitochondrial fragmentation.

Despite unravelling some novel mechanisms of cardiac injury under IH exposure in this study, several limitations pose the need for further investigations. First, the potential molecular pathways behind IH‐induced mitochondrial fission still remain unclear; thus, a great deal of work is needed to be performed. Second, only one dose of haemin was used in our animal study, whether haemin has a dose‐dependent protective effect on IH‐induced cardiac injury requires further investigation. Third, to further verify the suppressive effects of haemin on mitochondrial fission, interventional study performed with HO‐1 inhibitor (zinc‐protoporphyrin, ZnPP) should be carried out in the in vivo study.

In conclusion, our study demonstrated that IH induced functional and morphological heart abnormalities via mediating mitochondrial fission and cell apoptosis in both in vitro as well as in vivo model (Figure 7). Furthermore, our study provided the evidence that haemin exerted the protective effects on IH‐induced cardiac injury via the up‐regulation of HO‐1 to suppress mitochondrial fragmentation and cardiomyocyte apoptosis. Our results show that pharmacological modulation of HO‐1 pathway may offer a new therapeutic approach for OSA‐related cardiovascular diseases.

**Figure 7:** The proposed mechanisms involved in intermittent hypoxia‐induced heart dysfunction and the protective effect of haemin

## CONFLICT OF INTERESTS

The authors confirm that there are no conflict of interests.
